The article "SMARCB1 expression is a novel diagnostic and prognostic biomarker for osteosarcoma" was retracted in 2023. Reason: duplicated images.

# SMARCB1 expression is a novel diagnostic and prognostic biomarker for osteosarcoma

**DOI:** 10.1042/BSR20212446

**Published:** 2022-01-11

**Authors:** Tao Guo, Ran Wei, Dylan C. Dean, Francis J. Hornicek, Zhenfeng Duan

**Affiliations:** 1 Department of Gynecology and Obstetrics, West China Second Hospital, Sichuan University, Chengdu 610041, China; 2 Department of Orthopedic Surgery, Sarcoma Biology Laboratory, Sylvester Comprehensive Cancer Center, and The University of Miami Miller School of Medicine. Address: Papanicolaou Cancer Research Building, 1550 NW. 10th Avenue, Miami, FL 33136, U.S.A.; 3 Musculoskeletal Tumor Center, Beijing Key Laboratory of Musculoskeletal Tumor, Peking University People’s Hospital, No. 11 Xizhimen South Street, Xicheng District, Beijing 100044, China; 4 Department of Orthopaedic Surgery, Keck School of Medicine at University of Southern California (USC), USC Norris Comprehensive Cancer Center, 1441 Eastlake Ave, NTT 3449, Los Angeles, CA 90033, U.S.A.

**Keywords:** Biomarker, Immunohistochemistry, Osteosarcoma, Prognosis, Tissue microarray

## Abstract

**Background:** Although weak SWI/SNF related matrix-associated actin-dependent regulator of chromatin subfamily B member 1 (SMARCB1) expression is a known diagnostic and prognostic biomarker in several malignancies, its expression and clinical significance in osteosarcoma remain unknown. The aim of the present study was to investigate SMARCB1 expression in osteosarcoma and its clinical significance with respect to chemosensitivity and prognosis.

**Methods:** We obtained 114 specimens from 70 osteosarcoma patients to construct a tissue microarray (TMA) and assess SMARCB1 protein expression via immunohistochemistry (IHC). The mRNA expression of SMARCB1 was *in-silico* analyzed using open-access RNA sequencing (RNA-Seq) and clinicopathological data provided by the Therapeutically Applicable Research to Generate Effective Treatments on Osteosarcoma (TARGET-OS) project. The correlations between SMARCB1 expression and clinical features were statistically analyzed.

**Results:** Weak SMARCB1 expression occurred in 70% of the osteosarcoma patient specimens in the TMA, and significantly correlated with poor neoadjuvant response as well as shorter overall and progression-free survival (PFS). In addition, mRNA *in-silico* analysis confirmed that SMARCB1 expression correlates with chemotherapeutic response and prognosis in osteosarcoma patients.

**Conclusion:** To our knowledge, the present study is the first to analyze SMARCB1 expression in osteosarcoma. SMARCB1 may serve as a novel diagnostic and prognostic biomarker in osteosarcoma.

## Introduction

Osteosarcoma is the most common primary bone malignancy and most often occurs in children and adolescents [1,2]. Current treatment protocols typically utilize a combination of surgery and systemic neoadjuvant chemotherapy [3]. Although the 5-year survival rate for osteosarcoma patients has improved from 20 to over 65%, a considerable number of patients develop tumors which metastasize, locally recur, or evolve robust chemoresistance [4,5]. For these challenging cases, the 5-year overall survival (OS) rate decreases to a dismal 11–29% [6]. Because the molecular drivers initiating secondary osteosarcoma growths remain poorly defined, there has been an expansion of works seeking to identify predictive biomarkers. At present, however, the only accepted prognostic predictor for osteosarcoma patients is the percent necrosis of a resected tumor sample following neoadjuvant chemotherapy. However, its clinical utility in osteosarcoma has become increasingly controversial, and highlights the need for novel diagnostic and predictive biomarkers which may better predict and personalize therapy for osteosarcoma patients [7].

SWI/SNF related matrix-associated actin-dependent regulator of chromatin subfamily B member 1 (SMARCB1, also known as BAF47 or INI1) is a nuclear protein with a molecular mass of 47 kDa. It is the core component of the ATP-dependent SWI/SNF chromatin-remodeling complex, a protein which induces a nucleosome conformation more accessible to transcriptional machinery [8,9]. SMARCB1 has notable roles in epigenetic regulation, cell cycle progression, signaling cascade cross-talk, and transcription. Most importantly, SMARCB1 is a robust tumor suppressor gene with weak expression in various tumors, including various soft tissue and bone sarcomas [10–14]. There is, therefore, potential for SMARCB1 expression to serve as a diagnostic and prognostic biomarker [10–12,15–19]. Despite its well-documented significance in cancer treatment and detection, to our knowledge, the expression and clinical significance of SMARCB1 in osteosarcoma remain unknown.

The aims of the present study were to: determine the expression of SMARCB1 in osteosarcoma; identify whether a correlation exists between SMARCB1 expression and osteosarcoma response to neoadjuvant chemotherapy; and to investigate the correlation between SMARCB1 expression and osteosarcoma patient prognosis.

## Materials and methods

### Construction of the human osteosarcoma tissue microarray

A total of 114 formalin-fixed, paraffin-embedded (FFPE) osteosarcoma tissue specimen blocks were obtained from 70 enrolled patients to construct the tissue microarray (TMA). Informed consents were received from every osteosarcoma patient, of whom surgeries were performed from 1993 to 2010. All tissues were used in accordance with the policies of the Institutional Review Board (IRB) of the hospital and common rules of the U.S. Department of Health and Human Services as previously described [20,21]. The TMA was constructed by the Tissue Microarray and Imaging Core at the Dana-Farber/Harvard Cancer Center. To ensure that the selection included the core of the tumor tissues, and to avoid bias or variation with a tissue specimen, three sites of each FFPE block were selected for assembling the recipient master block. Representative triplicate 0.5-mm-diameter core biopsies of each tissue block were obtained through the pathology reports and reading of corresponding Hematoxylin and Eosin (HE)-stained slides by a pathologist, as we have reported previously [20,21]. Clinicopathological data of the specimens were collected from archives and included age, gender, disease status, neoadjuvant chemotherapy, tumor necrosis rate, and follow-up data (Table 1). Representative triplicate 0.5-mm-diameter core biopsies of each tissue block were confirmed by pathology reports to ensure inclusion of the tumor core. HE-stained slides from each tissue block were read by a pathologist. We categorized specimens into three groups according to patient disease status at the time of tumor sample obtainment: a primary group from patients with primary localized tumor without metastasis, a recurrence group from specimens of patients with recurrent tumor without metastasis, and a metastasis group from patients with metastatic lesions. Tumor necrosis data were obtained from the clinical data and grouped according to percent tumor tissue necrosis of the specimens. The specimens were subsequently divided into two groups according to response; good response: ≥ 90% necrosis; poor response: < 90% necrosis.

**Table 1:** Patient demographics and clinical data of the osteosarcoma TMA

Variable	Number (%) or mean value ± SD	
	Patients	Specimens
Number	70	114
Age	31.3 ± 17.2 years	
Gender		
Male	42 (60.0)	
Female	28 (40.0)	
Follow-up time	99.1 ± 80.2 months	
Disease status		
Primary	56 (80.0)	70 (61.4)
Recurrence	3 (4.3)	9 (7.9)
Metastasis	11 (15.7)	35 (30.7)
Neoadjuvant chemotherapy		
With	51 (72.9)	74 (64.9)
Good response (tumor necrosis rate ≥ 90%)	16 (31.4)	21 (28.4)
Poor response (tumor necrosis rate < 90%)	35 (68.6)	49 (66.2)
Without	19 (27.1)	40 (35.1)
Death	39 (55.7)	
Disease progression	44 (62.9)	

### Immunohistochemistry staining of the TMA

The expression of SMARCB1 was detected by immunohistochemistry (IHC) staining according to the manufacturer’s protocol (Cell Signaling Technology, Danvers, MA, U.S.A.). The TMA was deparaffinized with xylene three times for 5 min each, transferred through 100% ethanol twice for 5 min each, rehydrated through graded alcohol (100, 95, 70, and 50%, 5 min each), and finally immersed in deionized water for 10 min. Antigen retrieval was performed with Target Retrieval Solution (Dako North America, Inc., Carpinteria, CA, U.S.A.). Next, the slide was washed with phosphate-buffered saline (PBS) twice for 5 min each. Once antigen retrieval was complete, endogenous peroxidase activity was quenched by incubation in 3% hydrogen peroxide. Following protein blocking with blocking solution (Cell Signaling Technology, Danvers, MA, U.S.A.) for 1 h at room temperature, the slide was incubated with primary SMARCB1 antibody (1:50 dilution, Cell Signaling Technology, Danvers, MA, U.S.A.) at 4°C overnight in a humidified atmosphere. Each step was followed by three TBS rinses, and the bound antibody on the array was detected using SignalStain® Boost Detection Reagent (Cell Signaling Technology) and SignalStain® DAB (Cell Signaling Technology). Finally, the osteosarcoma sections were counterstained with Hematoxylin QS (Vector Laboratories), and the slide was mounted with VectaMount AQ (Vector Laboratories) for long-term preservation. Of note, no staining with SMARCB1 antibodies was appreciated in non-SMARCB1 expressing tissues.

### Evaluation of SMARCB1 via TMA immunostaining

For quantification of SMARCB1 expression, two independent investigators, blinded to patient data and tumor histopathological characteristics, viewed and scored the immunostained slides. Any differences in the scores were resolved by consensus after joint review of the slide and discussion between the two investigators. The nuclear immunostaining intensity pattern of SMARCB1 was semiquantitatively scored based on the percentage of cells showing positive nuclear staining: 0, no nuclear staining; 1+, <10% positive cells; 2+, 10–25% positive cells; 3+, 26–50% positive cells; 4+, 51–75% positive cells; 5+, >75% positive cells (Figure 1A). The weak expression group included specimens with 0 to 2+ staining, while the strong expression group included specimens with 3+ to 5+ staining. SMARCB1 staining images were obtained using a Nikon Eclipse Ti-U fluorescence microscope (Nikon Corp.) with a SPOTRT digital camera (Diagnostic Instruments, Inc.). The data on SMARCB1 expression were analyzed using GraphPad Prism 7.0 software (GraphPad Software Inc., San Diego, CA).

**Figure 1:** Immunohistochemical staining of SMARCB1 in a human osteosarcoma TMA (**A**) Representative images of different levels of SMARCB1 expression in osteosarcoma tissues: 0 to 2+ staining, weak expression; 3+ to 5+ staining, strong expression. (**B**) Distribution of SMARCB1 expression in osteosarcoma specimens. (**C**) Distribution of weak and strong expression of SMARCB1 in osteosarcoma specimens.

### Analysis of SMARCB1 expression from the public database

Genome-wide RNA sequencing (RNA-Seq) is a quantitative technique to detect changes of gene expression in tissues [22,23]. RNA-Seq data were obtained from an established public database and referenced to quantify SMARCB1 mRNA gene expression in osteosarcoma. The open access RNA-Seq data and corresponding clinicopathological information of the osteosarcoma samples were provided by Therapeutically Applicable Research to Generate Effective Treatments on Osteosarcoma (TARGET-OS, phs000468) at https://portal.gdc.cancer.gov/projects/TARGET-OS and downloaded from the UCSC Xena browser (https://xenabrowser.net). Transcripts per million unit (TPM) was used to compare gene expression from RNA-Seq [24].

### Statistical analysis

The data were analyzed using GraphPad Prism 7.0 software and SPSS 19.0 software (IBM Corp., Armonk, NY). Independent *t* tests, one-way analysis of variance (ANOVA), and Pearson correlation tests were used to compare SMARCB1 expression to clinicopathological features. OS and progression-free survival (PFS) were calculated using the Kaplan–Meier method. Log-rank tests were used to determine the differences of OS and PFS between different SMARCB1 expression levels. Prognostic factors associated with OS or PFS were analyzed using the Cox proportional hazards regression model. Results were presented as mean values and 95% confidence intervals (95% CIs) for survival analysis and mean ± SD for others. *P*-values <0.05 were considered statistically significant.

## Results

### Expression of SMARCB1 in osteosarcoma specimens

Among the 114 osteosarcoma patient specimens, nuclear immunostaining intensities varied from no staining (41, 36.0%) to 1+ staining (21, 18.4%), 2+ staining (18, 15.8%), 3+ staining (18, 15.8%), 4+ staining (11, 9.6%), and 5+ staining (5, 4.4%) (Figure 1B). According to the classification of staining intensity as described above in the ‘Materials and methods’ section, weak expression of SMARCB1 was found in 70.2% of all osteosarcoma specimens (Figure 1C).

The SMARCB1 expression levels in the osteosarcoma specimens were next analyzed according to disease status. Compared with primary group specimens, there was significantly lower SMARCB1 expression in the recurrence group (0.56 ± 0.88 versus 1.9 ± 1.6, *P*=0.01) and metastasis group (1.1 ± 1.3 versus 1.9 ± 1.6, *P*=0.008) (Figure 2A). We further examined SMARCB1 expression in specimens with advanced disease status (recurrence and metastasis), and found significantly weaker expression of SMARCB1 compared with specimens enrolled in the primary group (1.0 ± 1.2 versus 1.9 ± 1.6, *P*=0.001) (Figure 2B).

**Figure 2:** The correlation between SMARCB1 expression and disease status in osteosarcoma (**A**) Comparison of SMARCB1 expression level in specimens from primary, metastatic, and recurrent groups. (**B**) Comparison of SMARCB1 expression in specimens with primary and advanced disease status.

### Correlation of SMARCB1 expression to neoadjuvant chemotherapy response

A majority, 74 of the 114 (64.9%) specimens were treated with neoadjuvant chemotherapy, with the remaining 40 specimens (35.1%) having not undergone this treatment. Significantly decreased expression of SMARCB1 was seen in specimens without neoadjuvant chemotherapy compared with treated specimens (1.1 ± 1.3 versus 1.8 ± 1.6, *P*=0.015) (Figure 3A). Furthermore, among the 74 specimens treated with neoadjuvant chemotherapy, SMARCB1 expression was significantly weaker and there was comparatively poor chemotherapeutic response compared with specimens with a favorable response to neoadjuvant chemotherapy (1.5 ± 1.4 versus 2.7 ± 1.8, *P=*0.004) (Figure 3B). In addition, there was a significant correlation between SMARCB1 expression and tumor necrosis rate (Pearson r = 0.35, *P*=0.003) (Figure 3C).

**Figure 3:** The correlation between SMARCB1 expression and response to neoadjuvant chemotherapy in osteosarcoma (**A**) Comparison of SMARCB1 expression in specimens with and without neoadjuvant chemotherapy. (**B**) Comparison of SMARCB1 expression in specimens showing good and poor response to neoadjuvant chemotherapy. (**C**) The correlation between SMARCB1 expression and tumor necrosis rates in osteosarcoma specimens. (**D**) The comparisons of SMARCB1 expression between specimens with/without neoadjuvant chemotherapy and good/poor chemotherapeutic response in specimens obtained from patients with primary localized osteosarcoma. The numbers (*n*) in Figure 3A,B,D reflect the numbers of specimens of osteosarcoma blocks.

For the primary group, 24/70 specimens without neoadjuvant chemotherapy showed significantly attenuated SMARCB1 expression compared with the 46 specimens that underwent chemotherapy (1.3 ± 1.4 versus 2.3 ± 1.6, *P*=0.009). Among the 46 specimens with available tumor necrosis rate data, we found significantly decreased SMARCB1 expression in poor responders to neoadjuvant chemotherapy (31/46) compared with those with a favorable response (14/46) (1.8 ± 1.5 versus 3.4 ± 1.5, *P*=0.003) (Figure 3D).

### Correlation between SMARCB1 expression and patient OS

A total of 39 deaths occurred among the 70 patients in the follow-up period. Significantly weaker SMARCB1 expression was found in patients who died compared with those who were alive at the end of the follow-up period (1.4 ± 1.3 versus 2.9 ± 1.5, *P<*0.001) (Figure 4A).

**Figure 4:** The correlation between SMARCB1 expression and prognosis in osteosarcoma patients SMARCB1 expression was compared in patients who were dead or alive (**A**) and who had disease progression or were progression-free (**C**) at the endpoint of follow-up. Furthermore, in survival analysis, patients with strong SMARCB1 expression showed significantly better OS (**B**) and PFS (**D**) compared with patients with weak SMARCB1 expression.

The mean OS of the 70 osteosarcoma patients was 140.9 (95% CI: 113.2–168.6) months and the 5-year OS rate was 59.2% (95% CI: 47.4–71.0%). The 5-year OS rate of patients with weak SMARCB1 expression (45.5%, 95% CI: 30.0–61.0%) was significantly shorter than that in patients with strong SMARCB1 expression (78.9%, 95% CI: 63.8–94.0%) (*P*<0.001) (Figure 4B). The SMARCB1 expression underwent multivariate analysis alongside other factors in OS including age, gender, disease status, and response to neoadjuvant chemotherapy. The results of Cox regression confirmed that weak SMARCB1 expression was the only independent risk factor for shorter OS in osteosarcoma patients (*P*=0.015) (Table 2).

**Table 2:** Multivariate analysis of prognostic factors for osteosarcoma patient OS

Variable	HR	95% CI	*P*
Age			
≥27 yrs	0.87	0.39–2.0	0.74
<27 yrs			
Gender			
Male	0.60	0.27–1.3	0.21
Female			
Disease status			
Primary	0.59	0.25–1.4	0.23
Advanced			
Response to neoadjuvant chemotherapy			
Good	1.5	0.55–4.1	0.44
Poor			
SMARCB1 expression			
Strong	3.8	1.3–10.9	0.015^*^
Weak			

* Statistical significance. Abbrevitons: HR, hazard ratio; yrs, years.

### SMARCB1 expression and PFS in osteosarcoma patients

Among the 70 osteosarcoma patients in our sample, there were 51 disease-progressions during the follow-up period. Of note, SMARCB1 expression in patients with disease progression was significantly decreased compared to those without disease progression (1.5 ± 1.3 versus 3.0 ± 1.6, *P*<0.001) (Figure 4C).

The mean PFS was 112.4 months (95% CI: 85.2–139.6) and the 5-year PFS rate was 50.5% (95% CI: 38.3–62.7%). Patients with reduced SMARCB1 expression had significantly decreased 5-year PFS rates compared with patients with elevated SMARCB1 expression (35.3 versus 71.5%, *P*<0.001) (Figure 4D). Multivariate analysis for prognostic factors of PFS in osteosarcoma patients via Cox regression included SMARCB1 expression as well as age, gender, and response to neoadjuvant chemotherapy. Importantly, only weak SMARCB1 expression was an independent risk factor for PFS in osteosarcoma patients (*P*=0.011) (Table 3).

**Table 3:** Multivariate analysis of prognostic factors for PFS in 70 osteosarcoma patients

Variable	HR	95% CI	*P*
Age			
≥27 yrs	0.86	0.41–1.8	0.70
<27 yrs			
Gender			
Male	0.60	0.29–1.2	0.17
Female			
Response to neoadjuvant chemotherapy			
Good	1.4	0.57–3.5	0.46
Poor			
SMARCB1 expression			
Strong	3.1	1.3–7.4	0.011^*^
Weak			

* Statistical significance. Abbreviations: HR, hazard ratio; yrs, years.

### *In-silico* analysis between SMARCB1 gene expression and osteosarcoma clinicopathological features

SMARCB1 gene expression profiles and clinicopathological characteristics were available in TARGET-OS for 84 osteosarcoma samples. Twenty-one of the samples were from osteosarcoma patients with metastasis and 63 of the samples were from patients without metastasis. The SMARCB1 gene was poorly expressed in samples with metastasis compared with the non-metastatic samples (124.6 ± 56.8 versus 144.0 ± 60.1, *P*=0.20) (Figure 5A). Additionally, there were 43 available samples treated with neoadjuvant chemotherapy also having chemotherapeutic response data. Samples with poor response (<90% necrosis of tumor cells) to neoadjuvant chemotherapy showed reduced SMARCB1 gene expression compared with samples with good chemotherapeutic response (≥ 90% necrosis of tumor cells; 133.0 ± 66.7 versus 146.7 ± 58.4, *P*=0.49) (Figure 5B).

**Figure 5:** *In-silico* analysis of the correlation between SMARCB1 gene expression and clinicopathological characteristics of osteosarcoma patients using data obtained from the TARGET-OS project High SMARCB1 gene expression was observed in samples with no metastasis (**A**) and with good response to neoadjuvant chemotherapy (**B**). In survival analysis, patients with high SMARCB1 gene expression tended to show better OS (**C**) and PFS (**D**) compared with patients with low SMARCB1 gene expression.

We further performed a survival analysis of the clinical data for all 84 samples of osteosarcoma and found the mean OS and PFS in these patients were 98.9 months (95% CI: 84.6–113.1) and 76.6 months (95% CI: 61.3–92.0), respectively. Furthermore, the 5-year OS and PFS rates were 65.1% (95% CI: 53.7–76.5%) and 54.6% (95% CI: 43.2–66.0%), respectively. In both OS (70.5 versus 63.4% on 5-year OS rate, *P*=0.31) and PFS groups (71.4 versus 47.3% on 5-year PFS rate, *P*=0.074), the data showed a trend, although not statistically significant, towards worse clinical outcomes in patients with weak SMARCB1 gene expression (Figure 5C,D).

## Discussion

SMARCB1 is a well-known tumor suppressor in healthy cells, and when silenced, is highly tumorigenic [25]. Mechanistically, weak SMARCB1 expression is a result of gene mutation, deletion, or miRNA regulation in various cancers [11,26,27]. Loss of SMARCB1 impairs the function of the enhancers which facilitate cell differentiation, without affecting the so-called super-enhancers promoting undifferentiated cellular proliferation and tumorigenesis [28,29]. As expected, weak SMARCB1 expression has been recognized as a diagnostic biomarker in several tumors including epithelioid sarcoma, rhabdoid tumor, synovial sarcoma, and pediatric poorly differentiated chordoma [15,16,19]. In our study, weak SMARCB1 expression was seen in most osteosarcoma specimens, with absent expression occurring in nearly half of the specimens. When SMARCB1 expression was compared among specimens obtained from patients with variable disease status, we found weaker SMARCB1 expression is directly correlated with more advanced disease. We confirmed similar results at the gene expression level by *in-silico* analysis using mRNA-seq and clinicopathological data from the TARGET-OS project. Our findings are consistent with previous works that support the anti-tumorigenic role of SMARCB1 [14,27,30]. To our knowledge, this study is the first to show SMARCB1 expression as a potential prognostic biomarker and indicator of advanced disease status in osteosarcoma.

The application of chemotherapy, especially neoadjuvant chemotherapy, has become foundational for the treatment of osteosarcoma due to its dramatic and historic improvement in patient survival [4,5]. However, the major challenge to its effectiveness is the development of chemotherapeutic resistance in some patients. At present, the response to chemotherapy and the development of drug resistance are unpredictable by current screening tools. The sole marker for chemotherapeutic response in osteosarcoma is based on pathological analysis of the histological necrosis rate after neoadjuvant chemotherapy [31–33]. Previously, SMARCB1 and the SWI/SNF complex have shown to contribute to tumor chemosensitivity via facilitating decatenation of DNA by topoisomerase II [34]. Moreover, silencing of SMARCB1 can induce drug resistance by transcriptional up-regulation of the gene encoding multidrug resistance pump ABCB1 [35]. In a subsequent study, diminished SMARCB1 expression was shown to increase chemotherapeutic drug resistance in malignant cells [36]. Similarly, in our present work, we demonstrate weak SMARCB1 expression is associated with poor chemotherapeutic response in osteosarcoma. These findings are paralleled at the mRNA level by our *in-silico* analysis. Taken together, our results are consistent with previous works on SMARCB1 expression and drug resistance, suggesting that weak SMARCB1 expression may predict poor response to chemotherapy in osteosarcoma.

Several studies have also shown that decreased SMARCB1 expression is associated with poor prognosis in various tumors. In patients with colorectal cancer, loss of SMARCB1 expression is correlates with poor differentiation, liver metastasis, and shorter patient survival [17]. In a study on SMARCB1 expression in chordoma, loss of SMARCB1 was a marker for poor differentiation and dismal prognosis [37]. Furthermore, SMARCB1 expression is associated with pediatric chordoma prognosis, suggesting its utility for prognostic grading in this disease [18]. In our study, expression of SMARCB1 correlated with survival and disease progression for osteosarcoma patients. Furthermore, weak expression of SMARCB1 was an independent risk factor for OS and PFS in osteosarcoma. These results were also partially supported by *in-silico* survival analysis based on data from TARGET-OS, which showed a trend of weak SMARCB1 gene expression correlating with poor OS and PFS in osteosarcoma patients. The expression of SMARCB1 significantly correlated with patient survival in the TMA. Of note, there was also a trend, although not statistically significant, observed in the patient data from the TARGET-OS project. This discrepancy may reflect the differences in the patient samples. While most of the osteosarcoma tissue specimens obtained to construct the TMA in the present study were adult patients (average age: 31.3 years), the TARGET-OS project tissues were acquired from patients in studies and clinical trials managed through the Children’s Oncology Group (COG, patients were aged 14 years or less, https://ocg.cancer.gov/programs/target/projects/osteosarcoma). In addition, the TMA quantifies the protein level of SMARCB1 expression whereas the TARGET-OS dataset includes RNA level of SMARCB1 expression.

In summary, our study demonstrates weak SMARCB1 expression exists in most osteosarcoma tissues. Weaker SMARCB1 expression also correlates with poor response to neoadjuvant chemotherapy and is an independent prognostic risk factor in osteosarcoma. SMARCB1 is therefore a potential novel molecular diagnostic and prognostic biomarker in osteosarcoma.

## Data Availability

The data that support the findings of the present study are available from the corresponding author (Zhenfeng Duan) upon request.

## Abbreviations

FFPE: formalin-fixed, paraffin-embedded
HE: Hematoxylin and Eosin
OS: overall survival
PFS: progression-free survival
RNA-Seq: RNA sequencing
SMARCB1: SWI/SNF related matrix-associated actin-dependent regulator of chromatin subfamily B member 1
TARGET-OS: Therapeutically Applicable Research to Generate Effective Treatments on Osteosarcoma
TMA: tissue microarray
95% CI: 95% confidence interval
